# MeQryEP: A Texture Based Descriptor for Biomedical Image Retrieval

This article has been retracted.

**DOI:** 10.1155/2022/9505229

**Published:** 2022-04-11

**Authors:** G. Deep, J. Kaur, Simar Preet Singh, Soumya Ranjan Nayak, Manoj Kumar, Sandeep Kautish

**Affiliations:** ^1^Chandigarh Engineering College Landran, Mohali, India; ^2^Bennett University, Greater Noida, India; ^3^Amity School of Engineering and Technology, Amity University Uttar Pradesh, Noida, India; ^4^School of Computer Science, University of Petroleum and Energy Studies, Dehradun, India; ^5^LBEF Campus, Kathmandu 44600, Nepal

## Abstract

Image texture analysis is a dynamic area of research in computer vision and image processing, with applications ranging from medical image analysis to image segmentation to content-based image retrieval and beyond. “Quinary encoding on mesh patterns (MeQryEP)” is a new approach to extracting texture features for indexing and retrieval of biomedical images, which is implemented in this work. An extension of the previous study, this research investigates the use of local quinary patterns (LQP) on mesh patterns in three different orientations. To encode the gray scale relationship between the central pixel and its surrounding neighbors in a two-dimensional (2D) local region of an image, binary and nonbinary coding, such as local binary patterns (LBP), local ternary patterns (LTP), and LQP, are used, while the proposed strategy uses three selected directions of mesh patterns to encode the gray scale relationship between the surrounding neighbors for a given center pixel in a 2D image. An innovative aspect of the proposed method is that it makes use of mesh image structure quinary pattern features to encode additional spatial structure information, resulting in better retrieval. On three different kinds of benchmark biomedical data sets, analyses have been completed to assess the viability of MeQryEP. LIDC-IDRI-CT and VIA/I–ELCAP-CT are the lung image databases based on computed tomography (CT), while OASIS-MRI is a brain database based on magnetic resonance imaging (MRI). This method outperforms state-of-the-art texture extraction methods, such as LBP, LQEP, LTP, LMeP, LMeTerP, DLTerQEP, LQEQryP, and so on in terms of average retrieval precision (ARP) and average retrieval rate (ARR).

## 1. Introduction

Massive amounts of biomedical and health informatics data are generated on a regular basis as a result of the growth of biomedical imaging modalities, such as MRI, CT, ultrasound (US), and X-ray. A few investigations have reported the increment in imaging over time, yet generally little has been published about the characterizing patterns of imaging exhaustively. The primary goal here is to use such diverse biomedical imaging data and to develop new computational strategies so that a specialist can give an early analysis of the patients. Given that medical imaging is made of a variety of small structures, researchers have been particularly interested in developing well-structured approaches for working on large datasets of biomedical images for fast examination and retrieval. A deep learning technique for biomedical image identification and categorization on massive biomedical databases is used to find unpredictable patterns [1, 2]. The expertise of the content-based image retrieval (CBIR) technique is distributed to create content-based medical image retrieval (CBMIR) to solve the issue of biomedical images provided in comprehensive reviews [3–6]. In this context, it is found that the texture of the image provides useful discriminating visual feature information about the objects, content inside the image, and the connection with the background. Subsequently, the feature extraction of texture images has gotten perhaps the most challenging part in the processing of images using textural characteristics [7–9]. Local extreme co-occurrence patterns also played a vital role in texture analysis [10]. According to the perspective of directional characteristics-based texture retrieval, the patterns in three different orientations, such as diagonal, vertical, and horizontal, with discrete wavelet transform (DWT) are presented [11]. The appearance of any nodule/organ/lesion in clinical testing images is caused by changes in the intensity that affects different textural features. From that point, the texture turned out to be famous in the biomedical retrieval of images because of the significant importance of the texture obtained. With co-occurrence matrix, medical MRI and CT images' retrieval in different tissues is studied [12]. The motif co-occurrence matrix is used in the CBIR technique to outline texture characteristics [13]. Furthermore, textural information for retrieval of medical data with method of complexity was also analysed by using fractal dimension on various scaling factors [14]. The texture analysis is presented on the brain tumors dataset analysis [15]. By expanding GLCM to various scales based on Gaussian filtering, authors developed texture descriptors [16]. Yadav et al. [17] have suggested a compressive sampling-based technique for retrieving texture characteristics from big medical datasets. For the retrieval of content-based mammography, authors proposed techniques for texture features [18].

However, the computing complexity of the various methods employed based on the texture feature available in different literature is more expansive in terms of complexity [13, 15–17]. To overcome this complexity challenge, LBP suggested that it can be useful in various biomedical applications [19]. Furthermore, the same author executed more alterations, such as LBPriu2, LBPu2_P_R, GLBPu2_8_1, in LBP for texture characterizations because of its simplicity, very low computing complexity, ability to code small specifications, and resilience in detecting structural and textural information [20]. For image retrieval, BLK_LBP is proposed to utilize LBP characteristics to create block-based texture features [21]. To introduce the texture pattern approach, the extended form of the famous LBP feature is proposed, and the same can be termed as the center symmetric local binary pattern (CS-LBP) and local configuration pattern (LCP) texture descriptor [22, 23]. However, LCP and LBP descriptor are completely different [23]. Some of the other LBP versions are developed for texture image retrieval applications presented in the literature [24–26]. Other applications related to LTP and LBP [27, 28] have been explored, such as face classification [29]. Subsequently, a modified LBP suggested to obtain discriminative characteristics for the CBIR system was also presented [30].

To gain new texture features on biomedical images, rich literature on the extended algorithms of LBP, i.e., LTCoP [31], PVEP [32], GLMeP [33], DBWP [34], DLEP [35], LMEBP [36], LTrP [37], LQEP [38], LDEP [39], LDMaMEP [40], was studied. Previously, DLTerQEP [41], LMeTerP [42], and LQEQryP [42] proposed LBP moderation on biomedical datasets. Although we are already aware that LBP generates directional derivative first-order patterns, Zhang et al. suggested local derivative patterns (LDP) for facial identification and also investigated LBP as nondirectional local first-order patterns. Because of intensity variations, the appearance differentiation of individual objects in ordinary images is not detected by local binary and derivative pattern methods in the study of literature [43]. The LBP operator's primary drawback is that the limit of the binary function lies directly at the central pixel's intensity value, making it susceptible to noise. To address this flaw, the authors introduced LQP for texture analysis using two fixed thresholds specified by the user on medical images, which is one of the improved variants of LBP [44]. When compared to LBP, LQP has fewer pixel value variations [29]. By distinguishing the edges into more than three values, LQP has enhanced the performance of these techniques. To extract information from medical images, it employed a four-value code. In continuation to this, more discriminative features on biomedical datasets utilizing a nonbinary coding system, such as quinary coding rather than binary coding, were presented [45]. Furthermore, LQP was studied to extract the efficient features for indexing and retrieval [46]. Nanni et al. [47] have shown that combining texture descriptors with LQP and deep learning algorithms yields improved results on similar datasets used in the literatures. Rampun et al. [48] captured the texture information using the LQP operator for mammogram analysis. The local quinary pattern descriptor was compared to the most advanced texture descriptors [49]. In research by Rachdi et al. [50], the multiscale quinary pattern descriptor presented high capability over other local feature descriptors in extracting discriminative feature representation [50]. Ahmad et al. [51] investigated the use of a feature descriptor, i.e., directional local quinary patterns (DLQP) for detecting plant leaf diseases. In some more investigations, Murala and Jonathan [33] presented a technique called local mesh patterns (LMeP) for biomedical image retrieval that encrypts the gray scale connection among the close neighbors for a particular center pixel using three different orientations of mesh patterns. On different datasets, Rubavathi and Ravi [52] have used the LMCoP method for the retrieval of images. Until now, the typical LBP technique establishes a circumferential link between the referred pixel and its neighbors in the investigation. Rather than LBP, the LMeP technique establishes a link between a referred pixel's surrounding neighbors in an image. The number of neighbors has an impact on the possible relationships among them.

According to the research articles reviewed, despite the fact that LBP and its variations accomplish agreeable performance, a different technique to expand the discriminative power in biomedical images for better texture representation is required. Focusing on the further development of texture analysis performance, the local 2D patterns, traditional LBP, LQP, and LMeP texture methods encouraged us to form a practically simple yet strong approach, namely the quinary encoding on mesh patterns (MeQryEP), for the retrieval of biomedical images in this paper. The following are the major novelties of the proposed descriptor (MeQryEP): (a) it is, as of now, demonstrated by Tan and Triggs [29] and Zhu et al. [53] that the dependability of LTP and LBP is lowered for illumination changes, respectively. To resolve this issue, the possibility of LQP is utilized for representing biomedical images in the data sets. (b) It gathers quinary coding features from three different directional local mesh patterns in a given image, resulting in more spatial structure information and improved retrieval. (c) The proposed texture operator shows superior performance to many current advanced texture descriptors, and moreover, in view of its large discriminative power of texture features, it is more viable for the understanding and analysis of image texture.

The paper is prepared as follows: Section 1 gives a brief overview of medical image retrieval and associated research.  Section 2 also includes a brief discussion of local patterns and the suggested approach. The ideas of the proposed system framework and assessment measures are presented in Section 3. There are experimental findings and discussions in Section 4. Finally, in Section 5, concluding comments and some thoughts about the future are provided.

## 2. Examining Local Patterns and Proposing a Novel Method

Here, we will go through a few of the most common texturing techniques that have been described in the literature. Given its ease-of-implementation consideration, the decision is centered on the usage of a block of 3 × 3 size, which is considerably the most necessary neighborhood, particularly in real-time applications.

### 2.1. Primary Version: Local Binary Patterns (LBPs)

The LBP operator developed by Ojala et al. is the most effective and frequently used local texture descriptor [20]. LBPs are resistant and durable to the constant changes in intensity in their original and improved forms because of their discriminative power, simple implementation, and low computational complexity. Hence, many researchers have considered it. By threshing the intensity of the adjacent pixels, the LBP technique describes the local contrast and spatial structure of each 3 × 3 local area in the image. Given a n × m pixels gray scale image *I*, where *I* (g) indicates the gray level of the image's g th pixel. At each pixel, the LBP operator is generated by comparing the binary value differences around the value of a central pixel, g_c_, in a small rounded neighborhood (with radius R). The current pixel's value of LBP is calculated as follows:

(1) $$\begin{array}{c} {\text{LBP}}_{\text{P},\text{R}}=\overset{\text{P}-1}{\underset{\text{p}=0}{\sum }}{\text{f}}_{1}\left({\text{g}}_{\text{p}-}{\text{g}}_{\text{c}}\right)2^{\text{p}},{\text{ f}}_{1}\left(\text{x}\right)=\left\{\begin{array}{cc} 1, & if\;x\geq 0,\\ 0, & \text{otherwise}, \end{array}\right) \end{array}$$

where

 
g_c_: center pixel's gray value
   g_p_: the gray symmetric circular values of neighborhood, g_p_ (*p* = 0,..., *P* − 1).
   P: pixels of image in the radius circle R(*R* > 0
   2^p^: factor of binomial for each sign f_1_ (g_p−_g_c_)

After determining the LBP value of each pixel in the image, a histogram is created to characterize the texture image.  Figure 1 displays a circular neighborhood set example for various patterns of (P, R).

### 2.2. Local Quinary Patterns (LQPs)

Nanni et al. introduced another variation of LBP for the analysis of the medical image, using a quinary encoding termed LQP in the elliptical neighborhood [44]. The difference between the center pixel's gray value and the gray values of one of their neighbors in this variation assumes 5-digit encryption values (i.e., −2, −1, 2, 1, and 0) rather than the 02 values (i.e., 1, 0) or 03 values (i.e., −1, 1, and 0) in the normal LBP and LTP. The code of binary LBP is substituted by a code of quinary LQP, and the indicator *f*_1_(x) is substituted with a 05-valued function based on two thresholds, t_1_ and t_2_, stated in equation (2).

(2) $$\begin{array}{c} {\overset{↔}{{\text{f}}_{1}}\left(\text{x},{\text{t}}_{1},{\text{t}}_{2}\right)=\left\{\begin{array}{cc} +2, & x\geq {\text{g}}_{\text{c}}+{\text{t}}_{2},\\ +1, & {\text{g}}_{\text{c}}+{\text{t}}_{1}\leq x<{\text{g}}_{\text{c}}+{\text{t}}_{2},\\ 0, & {\text{g}}_{\text{c}}-{\text{t}}_{1}\leq x<{\text{g}}_{\text{c}}+{\text{t}}_{1}\\ -1, & {\text{g}}_{\text{c}}-{\text{t}}_{2}\leq x<{\text{g}}_{\text{c}}-{\text{t}}_{1},\\ -2, & \text{otherwise}. \end{array}\right|}_{\text{x}={\text{g}}_{\text{p}}}, \end{array}$$

The subsequent binary function b_c_(x),  c ∈ {−2,   − 1, 1,  2} is used for conversion in equation (3).

(3) $$\begin{array}{c} {\text{b}}_{\text{c}}\left(\text{x}\right)=\;\left\{\begin{array}{cc} 1, & x=c,\\ 0, & \text{otherwise}. \end{array}\right) \end{array}$$

When *c* = 1, *c* = −1, *c* = −2, and *c* = 2 are used, the 1^st^ binary pattern is formed. The 2^nd^, 3^rd^, and 4^th^ binary coding patterns are produced in the same way. Finally, from these, four binary patterns' histograms are constructed. After that, 04 histograms are combined to obtain features.  Figure 2 shows an illustration of the patterns of the quinary [44] being divided into 04 binary patterns.

### 2.3. Local Mesh Patterns (LMeP)

The LMeP for the retrieval of biomedical images is designed by Murala and Jonathan using the LBP concept [33]. The LMeP value is calculated using the surrounding neighbors' relationship for a particular center pixel in the image [see in (equation (4))].

(4) $$\begin{array}{c} {\text{LMeP}}^{\text{j}}{}_{\text{P},\text{R}}=\overset{\text{P}}{\underset{\text{i}=1}{\sum }}2^{\left(\text{i}-1\right)}\times {\text{f}}_{1}\left({{\text{g}}_{\varphi }|}_{\text{R}}-{{\text{g}}_{\text{i}}|}_{\text{R}}\right),\\ \;\varphi =\text{1}+\text{mod}\left(\left(\text{i}+\text{P}+\text{j}-1\right)\text{,P}\right),\\ \forall \text{j}=1\text{, }2\text{,}..\text{,}\left(\text{P}/2\right), \end{array}$$

where *j* is the LMeP index, and the x/y operation's remainder is given by mod (*x*, *y*).

The potential LMeP patterns (particular 3 × 3 pattern) (LMeP_8_1, LMeP_16_2, LMePu2 (with uniform patterns)) for the P neighbors are P/2, and in this study, we exclusively experiment with the first 03-oriented LMeP patterns for *j* = 1, 2, 3 in equation (4), as shown in Figure 3. Next, the extended local mesh ternary pattern (LMeTerP) descriptor (Deep et al. [42]), where the LTP (Tan and Triggs [29]) connection is between the center pixel (gray value “16”) and neighbors (at threshold, *t* = 2) for the first mesh pattern image, is also shown in Figure 4. From the ternary pattern {−1, −1, −1, −1, −1, 1, −1, −1}, the upper LTP and lower LTP are converted. The unique LMeTerP values are calculated from LTP patterns. Other mesh pattern images had their LMeTerP values computed as well. The LBP and the initial 03 LMeP for a specified (P, R) [(8, 1), (16, 2), and (24, 3) for experimentation] with the center pixel (gray value “16”) highlighted in green color and the computations and the LMeTerP calculations of that local mesh patterns are shown in Figure 4.

### 2.4. Proposed Method: Quinary Encoding on Mesh Patterns (MeQryEP)

In this paper, the concept of local pattern techniques (LBP, LMeP, and LQP) has been used to state MeQryEP. With three mesh pattern orientations, MeQryEP describes the gray scale connection among the surrounding neighbors for a particular center pixel. It uses quinary pattern features from image mesh structures to obtain extra spatial structure information. Because of the five encoding techniques that create more texture patterns, its extracted features are more robust than other approaches, such as LBP, LTP, and other advanced texture descriptors.

We used the given image's convolution operations (see equations (2) & (4)) to produce the 03 images each of the local mesh pattern for *j* = 1, 2, 3 to expand the conventional LQP to MeQryEP.

(5) $$\begin{array}{c} {\text{MQryP}}_{\text{P,R}}^{\text{j}}=\text{conv}2\left({\text{LBP}}_{\text{mesh}},\text{win}\_\text{dir}\_\text{vec}\left\{1,\text{j}\right\}{,}^{\prime }\text{sam}e^{\prime }\right);\forall \text{j}=1\text{ to }\left(\left(\text{P}/2\right)-1\right). \end{array}$$

where LBP_mesh_: [Npixels(:, 1:P), Npixels(:, 1:P)]. The neighboring pixels' array of the given image (I) is represented by Npixels (P, R).

win_dir_Vec: A directional padding vector for windows that move over LBP_mesh_. Window(win_dir_vec) with (*j* = 1, 2, 3) is as follows: win_dir_vec {1, 1}, win_dir_vec {1, 2} ,  win_dir_vec {1, 3}, according to the five values (−2,   − 1,  0 ,  1,  2) of the quinary coding.

  ‘Same': the central portion of a convolution that is the same size as LBP_mesh_.

Equation (5) yields a five-value code array with the values (−2/−1/0/1/2). Using the idea of LQP provided, the produced mesh quinary pattern is further transformed into 04 binary coding patterns (upper and lower LQP coding patterns) at different thresholds (*t*_1_, *t*_2_). The unique MeQryEP values (decimal values) are also defined by a binomial weight multiplied with each LQP coding for a specific mesh pattern image selected (3 × 3) for the characterization of local pattern spatial structure. Two higher LQP (for *c* = 2 and 1 as in equation (3)) equations are defined as below in equations (6) and (7).

(6) $$\begin{array}{c} {\text{MQryP}}_{\text{upper}1}\left(1,\text{ j}\right)=\overset{\left(\text{P}/2\right)-1}{\underset{\text{j}=1}{\sum }}\overset{⟶}{{\text{f}}_{2}}\left(\text{x},{\text{ t}}_{1},{\text{t}}_{2}\right)\times 2^{\text{j}-1}, \end{array}$$

where $\overset{⟶}{{\text{ f}}_{2}}\left(\text{x},{\text{ t}}_{1},{\text{t}}_{2}\right)=\;\left\{\begin{array}{cc} 1\text{,} & if\left(\text{x}\geq {\text{t}}_{2}\right),\\ 0, & \text{otherwise}. \end{array}\right)$

(7) $$\begin{array}{c} {\text{MQryP}}_{\text{upper}2}\left(1,\;3+\text{j}\right)=\overset{\left(\text{P}/2\right)-1}{\underset{\text{j}=1}{\sum }}\overset{⟶}{{\text{f}}_{2}}\left(\text{x},{\text{ t}}_{1},{\text{t}}_{2}\right)\times 2^{\text{j}-1}, \end{array}$$

where $\overset{⟶}{{\text{ f}}_{2}}\left(\text{x},{\text{ t}}_{1},{\text{t}}_{2}\right)=\left\{\begin{array}{cc} 1, & if\left({\text{t}}_{1}\leq \text{x}<{\text{t}}_{2}\right),\\ 0, & \text{otherwise}. \end{array}\right)$

Similarly, (for *c* = −1 and −2 as in equation (3)), two lower LQP equations ((8) and (9)) are computed as follows:

(8) $$\begin{array}{c} {\text{MQryP}}_{\text{lower}1}\left(1,7+\text{j}\right)=\overset{\left(\text{P}/2\right)-1}{\underset{\text{j}=1}{\sum }}\overset{⟶}{{\text{f}}_{2}}\left(\text{x},{\text{ t}}_{1},{\text{t}}_{2}\right)\times 2^{\text{j}-1}, \end{array}$$

where

(9) $$\begin{array}{c} \overset{⟶}{{\text{ f}}_{2}}\left(\text{x},{\text{ t}}_{1},{\text{t}}_{2}\right)=\left\{\begin{array}{cc} 1, & if\left({\text{t}}_{1}\leq \text{x}<{\text{t}}_{2}\right),\\ 0, & \text{otherwise}, \end{array}\right.\\ {\text{MQryP}}_{\text{lower}2}\left(1,10+\text{j}\right)=\overset{\left(\text{P}/2\right)-1}{\underset{\text{j}=1}{\sum }}\overset{⟶}{{\text{f}}_{2}}\left(\text{x},{\text{ t}}_{1},{\text{t}}_{2}\right)\times 2^{\text{j}-1}, \end{array}$$

where

(10) $$\begin{array}{c} \overset{⟶}{{\text{ f}}_{2}}\left(\text{x},{\text{ t}}_{1},{\text{t}}_{2}\right)=\;\left\{\begin{array}{cc} 1\text{,} & if\left(\text{x}\geq {\text{t}}_{2}\right),\\ 0, & \text{otherwise}. \end{array}\right) \end{array}$$

A range of values from (0 to 2P-1) is of each of MeQryEP method, LQP (01 upper and 01 lower LQPs) map of the mesh images. Following the detection of local patterns, (LBP, MQryP, LQP, or MeQryEP) constructs a final histogram feature vector (by concatenating four descriptor histograms of each LQP operator) using the following equation (10).

(11) $$\begin{array}{c} {\text{H}}_{\text{MeQryEP}}\left(\text{v}\right)=\frac{1}{{\text{k}}_{1}\times {\text{k}}_{2}}\overset{{\text{k}}_{1}}{\underset{\text{q}=1}{\sum }}\overset{{\text{k}}_{2}}{\underset{\text{r}=1}{\sum }}{\text{f}}_{3}\left(\text{MeQryEP}\left(\text{q},\text{r}\right),\text{v}\right),\\ \text{v}\in \left[0,\;\left(2^{\wedge }\text{P}-1\right)\right],\\ {\text{f}}_{3}\left(\text{x},\text{y}\right)=\left\{\begin{array}{cc} 1, & \;if\left(\text{x}=\text{y}\right),\\ 0, & \;if\left(\text{x}\neq \text{y}\right), \end{array}\right)\; \end{array}$$

where an input image's size is represented by *k*1 × *k*2.

As we know, the high number of feature dimensions (from 2P to 5P) affects LQP, thus summing the retrieved patterns, as seen in equation (2), which is a good idea (using 5-value quinary F coding). Nanni et al. handled the above-mentioned difficulty by dividing each quinary pattern code into 04 binary patterns scheme (02 upper LQPs and 02 lower LQPs) in this study utilizing two user thresholds (t_1_, t_2_) (see in equations (5) to (9)) [44]. The original LQP operator is inferior because of its splitting into 02 LBPs on the upside and 02 on the downside. This study explores the optimum performance with a suitable feature dimension. In local mesh patterns, an illustration of MeQryEP computation for center pixel (the gray value “16”) highlighted in the green color is shown in Figure 5. Look at the initial MeQryEP mesh pattern image. As a result of equation (4), the neighbors are {57, −11, 12, −9, −15, −54, 62, −42}. The obtained result replaces the five-valued function $\;\overset{↔}{{\text{f}}_{1}}\left(\text{x},{\text{t}}_{1},{\text{t}}_{2}\right)$ (as in equation (2)) on the thresholds (*t*1 = 3, *t*2 = 7), and we obtain {2, −2, −1, −2, −2, −2, 2, −2} quinary values (tolerance of center pixel values are 16 ± 3 for t1 and 16 ± 7 for t2). Using equations (5) to (9), the quinary value coding is transformed into 04 binary patterns, such as upper LQPs and lower LQPs. Finally, the weights are added to each pattern, yielding 04 distinct values (42, 0, 0, 213) that are pointed to MeQryEP for the characterization of the local pattern's spatial structure. In addition, MeQryEP values for various mesh pattern images will be computed. The reason for that is the proposed descriptor results in more spatial structure information, improved retrieval, and also high performance because of its large discriminative power of texture features.

The proposed MeQryEP is different from the earlier acquainted, existing technique of LBP. With three specified orientations of mesh patterns, MeQryEP extracts the gray scale connection for a given center pixel among the neighbors, while LBP mines the gray scale connection between a center pixel and its neighbors' pixels. MeQryEP uses quinary pattern features from the mesh structures of an image to get extra information of the spatial structure that makes it different from the previously used LBP. It helps in the identification of the descriptive features of biomedical images using more discriminating code than binary and a pool of thresholds.

The LBP, LTP, and MeQryEP replies in a facial reference image are illustrated in Figure 6. Face image is used since it gives visually understandable results to distinguish the efficacy of various techniques. The feature map of the texture technique MeQryEP (upper and lower LQPs) captures more directional edge information than the LBP and LTP feature map for the extraction of texture.

## 3. Extraction of Features and the Proposed Method's Framework

### 3.1. Extracting Features

The process for the feature extraction using MeQryEP is demonstrated in Figure 7, and the stepwise approach is described below.

  (Input): image query as an input
  Output: retrieval results as the output
(1) Open an image that you are looking for (or gray-scale image): query image
(2) Form local mesh pattern designs at (*j* = 1, *j* = 2, *j* = 3) amongst the neighbors for a given central pixel.
(3) For each mesh pattern, calculate the MeQryEP quinary coding at various thresholds values (t1, t2) and adjust the *t* values as necessary.
(4) Split each quinary coding into 04 binary patternsl, such as upper LQPs and lower LQPs.
(5) For upper and lower LQPs, compute MeQryEP decimal values.
(6) Make a histogram for each binary pattern.
(7) Concatenate the histograms to create a feature vector.
(8) For comparing query image with a database image, (12) is employed.
(9) The images will be returned based on the finest matches.

### 3.2. A Measure of Similarity

This is a representation of the feature vector's query image, obtained by extracting the feature f_Q_=(f_Q_1__, f_Q_2__,…,  f_Q_L_g___). Also, the |DB| dataset of each medical image is provided with feature vectors f_DB_j__=(f_DB_j1__, f_DB_j2__,…,  f_DB_jL_g___); j=1,2,…,  |DB|. The only aim is to retrieve *n* top match images in the |DB| dataset by the measurement of the distance between the query image and the image of the dataset. The *n* finest images comparable to the query image will finally appear.

For the purposes of measuring similarity distance, the following D metric is employed:

(12) $$\begin{array}{c} \text{D}\left(\text{Q},\text{DB}\right)=\overset{{\text{L}}_{\text{g}}}{\underset{\text{i}=1}{\sum }}\left|\frac{{\text{f}}_{{\text{DB}}_{\text{ji}}}-{\text{f}}_{\text{Q},\text{i}}}{1+{\text{f}}_{{\text{DB}}_{\text{ji}}}+{\text{f}}_{\text{Q},\text{i}}}\right|, \end{array}$$

where the i^th^ feature of the j^th^ image in the dataset |DB| is f_DB_ji__.

### 3.3. The Framework of the Proposed System

Figure 8 shows the suggested system retrieval framework flowchart utilizing MeQryEP.

### 3.4. Measures of Assessment

Average precision, precision, average retrieval precision (ARP), average recall, recall, and average retrieval rate (ARR)), as computed by equations (12) to (15), are the measurements for the performances of the suggested technique. The precision (P) and recall (*R*) for query image, Iq, have the following definitions:

(13) $$\begin{array}{c} \text{Precision}:\text{P}\left({\text{I}}_{\text{q}}\right)=\;\frac{\text{Number of relevant images retrieved}}{\text{Total number of images retrieved}}. \end{array}$$

(14) $$\begin{array}{c} \text{ARP}=\frac{1}{\left|\text{DB}\right|}\overset{\left|\text{DB}\right|}{\underset{\text{i}=1}{\sum }}\text{P}{\left({\text{I}}_{\text{i}}\right)|}_{\text{n}\leq 10}. \end{array}$$

(15) $$\begin{array}{c} \text{ Recall}:\text{R}\left({\text{I}}_{\text{q}}\right)=\;\frac{\text{Number of relevant images retrieved}}{\text{Total number of relevant images in the database}}. \end{array}$$

(16) $$\begin{array}{c} \text{ARR}=\frac{1}{\left|\text{DB}\right|}\overset{\left|\text{DB}\right|}{\underset{\text{i}=1}{\sum }}{\text{R}\left({\text{I}}_{\text{i}}\right)|}_{\text{n}\geq 10}. \end{array}$$

## 4. Findings from the Experiments and Discussions

Experiments on three distinct medical datasets are used to access the performance of the suggested method employing nonbinary enlargement, such as quinary coding for the retrieval of biomedical images. The suggested method's findings are evaluated in the subsections that follow.

Every image in the database is picked as a query image in each trial. The system gathers *n* images of database X=(x_1 _,  x_2_,   …  ,  x_n_) for each query, with the smallest image matching distance (equation (12)). We may conclude that the system has properly matched if and only if the required series (x_i_;  *i* = 1, 2,...,*n*) are related to the same class of the query image. We investigated the influence of a collection of alternative pairs of thresholds (t_1_, t_2_) (upper and lower thresholds) in this research since we know that threshold selection is a vital task. Equations (5) to (9) are used here to calculate quinary values on these sets of pairs of thresholds. To extract a distinct feature set according to a pair of thresholds and select the dataset optimized thresholds that give the best retrieval results with respect to ARP and ARR on given different three biomedical datasets, a group of different threshold pairs according to t_1_={1,…, 25} and t_2_={t_1_+2,…, 27} are chosen.

### 4.1. LIDC-IDRI-CT (Dataset 1) Experiment

The dataset consists of 84 instances, each with around 100–400 images of digital imaging and communication (DICOM) and an XML data file, including the physician annotations. This dataset is the public CT scan image database (lung image database consortium and image database resource initiative (LIDC-IDRI) by Kascic and NEMA-CT online image database that is used for experimentation [54, 55]. There are 143 nodules in the database, ranging in size from ≤3 to ≥ 30 mm (separated physically by radiologists). LIDC 2 image toolkit (accessible online, Lampert) converts the CT lung imaging (512 × 512) into the “tif” imagery image format of the database for fast execution [56]. It was the radiologists' job to find the nodule sites, and they were given a list of 12 patients with a total of 75 nodules (26 benign and 49 malignant) and 229 slices. Additionally, the regions of interest (ROIs) were manually marked from each slice of certain patients to create the database of ROI CT images.  Table 1 lists the details of the CT scan data collection. The sample nodule lung images from the lung database are shown in Figure 9 (one image from each patient scan).

As illustrated in Figure 10 and Table 2, the suggested method's performance is measured with respect to ARR and ARP. By passing various query images (i.e., 1–10) on the dataset 1, Figure 10 demonstrates the performance retrieval of the given proposed approach (MeQryEP) and some other current approaches (LBPu2, LBPriu2, LQP, DLTerQEP, LMeP, LMeTerP, LQEQryP) with respect to ARR and ARP. The circular neighborhoods (8, 1) and (16, 2) are used in set for different (P,R) of LBP with uniform patterns. On the dataset 1, the suggested technique (MeQryEP) is evaluated for quinary value computation with two distinct thresholds (t_1_, t_2_). It has been noted that the thresholds (3, 7) function better for MeQryEP with respect to ARR. Table 2 highlights the performance of several approaches. In the majority of situations, MeQryEP outperforms the current techniques LBPu2, LBPriu2, LQP, DLTerQEP, LMeTerP, and LQEQryP, as shown in Figure 10. Three query results of the suggested technique (MeQryEP) based on ten top matches on the given dataset are shown in Figure 11.

### 4.2. VIA and I-ELCAP-CT (Dataset 2) Experiment

Public collection of vision and image analysis group (VIA) and international early lung cancer action program (I-ELCAP) provided a computer tomography (CT) dataset to evaluate several computer-aided detection methods (online access from VIA/I-ELCAP CT (dataset (2) lung image dataset) [57]. DICOM format is used to store these images. The thickness of a 1.25-mm slice can be obtained in a single breath hold with CT scans. They were also told the sites of nodules found by radiologist. As a result, the ROI CT image database is created using ROIs that have been manually annotated.  Table 3 displays the results of the tests on the date acquisition information of 10 CT scans with 100 images each and a resolution of 512 × 512. Dataset 2 sample images are shown in Figure 12 (one image from each category).

With respect to ARR and ARP, Figure 12 compares the performance retrieval of the suggested approach (MeQryEP) with that of other current methods ((LBPu2, LTP, LDP, LTCoP, PVEP, LTrP, LMeP, LMePu2, LQEP, DLTerQEP, LMeTerP, and LQEQryP). The circular neighborhoods (8, 1) and (16, 2) are used in set for different (P, R) of LBP with uniform patterns. On the dataset 2, the suggested technique (MeQryEP) is evaluated for quinary value computation with two distinct thresholds (t_1_, t_2_). It has been detected that the thresholds (2, 23) function better for MeQryEP. In terms of recall, Table 4 demonstrates group-based performance in the dataset 2 of the suggested approach and additional current methods.  Figure 13 shows the performance of each category with respect to recall and precision of the approach suggested, as well as other current approaches. On the dataset 2, the suggested approach (MeQryEP) clearly outperforms other current methods with respect to ARP, ARR, precision, and recall, as shown in Figures 13 and 14.

### 4.3. OASIS-MRI (Dataset 3) Experiment

The open access series of imaging studies (OASIS) dataset is used in the experiment. The open access imaging series was established by Marcus et al. and represents an advance of magnetic resonance imaging (MRI) data (dataset for usage in the medical research sector is available online) [58]. Specifics of the MRI acquisition are given in Table 5. Four hundred and twenty-one patients ranging in age from 18 to 96 are included in this data set. In addition, four categories (124, 102, 89, and 106 pictures) are classified in 421 images to test the retrieval of images based on the form of the ventricle in the images.  Figure 15 shows one sample image from each dataset 2 type.

With respect to ARP, Table 6 highlights the retrieval outcomes of MeQryEP and additional current techniques on the OASIS dataset. With respect to ARP (i.e., at *n* equal to10) in Table 6 and Figure 16, the following conclusions are drawn:

When compared to other retrieval methods (LBPu2_8_1 (41.8%), LDP (41.26%), LTP (44.44%), BLK_LBP (43.63%), CS_LBP (41.06%), LMEBP (43.08%), PVEP (45.71), LTrP (42.25%), LQEP (40.51%), LMePu2_8_1 (44.24%), GLBPu2_8_1 (41.23%), DLTerQEP (45.11%), LMeTerP (45.62%), and LQEQryP (46.23%)), the suggested directional pattern approach (MeQryEP (46.78%) has a better average retrieval precision.

Graphs illustrating the performance retrieval of the suggested approach and additional current methods with respect to ARP in accordance with the number of highest matches are shown in Figure 16(a). On the OASIS-MRI image database, Figure 16(b) shows the group-wise performance of several techniques with respect to ARP. On the OASIS-MRI dataset, the suggested technique (MeQryEP) is tested for the quinary value computation with two distinct thresholds (t_1_, t_2_). It can be shown that the thresholds (11, 13) perform better for MeQryEP. It is evident from Figure 16 that the suggested technique exceeds a large number of other current methods for the biomedical image retrieval of OASIS-MRI image databases.

### 4.4. Performance of Feature Vector Size

Using LBP, LTP, LDP, LTCoP, PVEP, LTrP, DLEP, LMeP, LQEP, LMeTer, DLTerQEP, and LQEQryP, Table 7 lists the feature vector size for a particular query image. The testing is done on Intel core i3-10th Gen processor, 4 GB of memory, and 256 GB SSD. The MATLAB Simulink is used to implement all of the techniques. Table 7 makes it obvious that the suggested approach's (MeQryEP) vector length is larger in comparison to some other current techniques, as it exceeds three distinct biomedical databases with regard to ARP and ARR.

## 5. Conclusions and Prospects for the Future

Here, a conceptually simple, easy-to-implement, and highly discriminating texture operator named “MeQryEP” is designed for the indexing and retrieval of the biomedical image based on various state-of-the-art techniques, such as LBP (LQP, LMeP, and LMeTerP), which are so-calling mesh pattern encoding. The approach suggested codes for the connection between the gray scale of a given center pixel for the neighboring areas with three specified mesh pattern orientations. The core of the approach is to encrypt additional information about spatial structure using quinary patterns from the mesh image structures. The findings of three distinct types of medical databases are taken to evaluate the strength and efficacy of the novel nonbinary coding technique. MeQryEP demonstrated its high capability, with great accuracy, to discriminate between LBP, LTP, LQEP, LMeP, LMeTerP, DLTerQEP, LQEQryP, and additional current state-of-the-art techniques on used LIDC-IDRI-CT, VIA/I-ELCAP-CT, and OASIS-MRI benchmark texture datasets, as demonstrated by its test results. Furthermore, this work can be valuable in the different uses of indexing and recovery of images based on content. In the future, the experimentation should likewise be possible utilizing other well-known nonbinary coding schemes like octal coding to increase the retrieval of the proposed technique performance. Three distinct types of benchmark biomedical databases are used to assess the appropriateness of the suggested descriptor. The suggested descriptor may be compared with the most advanced descriptors and evaluated on hundreds of biomedical datasets, including Covid-19 variant datasets. Execution time can also be considered to be a performance parameter in the future.

## Figures and Tables

**Figure 1:** Circular neighborhood sets for different (P, R).

**Figure 2:** Calculation of LBP and LQP operators.

**Figure 3:** The LBP and the first three LMeP calculations for a given (P, R) [33].

**Figure 4:** Example of obtaining LBP and LMeTerP for the 3 × 3 pattern [42].

**Figure 5:** Example to obtain MeQryEP calculation for the 3 × 3 pattern of an image at (*P* = 8, *R* = 1).

**Figure 6:** Response of proposed method on a reference face.

**Figure 7:** Procedure of feature extraction for MeQryEP.

**Figure 8:** Flowchart of the proposed retrieval system framework.

**Figure 9:** Sample nodule images from LIDC-IDRI-CT image database.

**Figure 10:** Performance comparison of the proposed method (MeQryEP) with other existing methods by passing different query images (1–10) in terms of (a) ARP and (b) ARR on LIDC-IDRI-CT database.

**Figure 11:** Query results of MeQryEP on LIDC-IDRI-CT database by passing three query images (a–c).

**Figure 12:** Sample images from VIA/I-ELCAP-CT image database.

**Figure 13:** Category-wise performance of MeQryEP and other existing methods in terms of (a) precision and (b) recall on VIA/I-ELCAP-CT database.

**Figure 14:** Comparison of the MeQryEP with other existing methods in terms of (a) ARP and (b) ARR on VIA/IELCAP-CT database.

**Figure 15:** Sample images from OASIS-MRI database.

**Figure 16:** (a) Comparison of the proposed method with other existing methods on different values of (P, R) as a function of the number of top matches and (b) different group of images (based on the shape of ventricular in the images) comparison of the proposed method with other existing methods on the OASIS-MRI database.

**Table 1:** Data acquisition details of LIDC-IDRI-CT image database.

Case no.	Data	No. of slices	No. of images	Resolution	Slice thickness (mm)	Tube voltage (kv)	Tube current (mA)
1	LIDC-IDRI-0002	20	40	512 × 512	1.3	120	440
2	LIDC-IDRI-0003	10	40	512 × 512	2.5	120	300
3	LIDC-IDRI-0006	20	80	512 × 512	1.3	120	440
4	LIDC-IDRI-0007	21	84	512 × 512	1.3	120	440
5	LIDC-IDRI-0010	15	60	512 × 512	1.3	120	401
6	LIDC-IDRI-0011	27	108	512 × 512	2.5	120	265
7	LIDC-IDRI-0012	20	80	512 × 512	2.5	120	300
8	LIDC-IDRI-0013	18	72	512 × 512	2.5	120	320
9	LIDC-IDRI-0014	07	28	512 × 512	2.5	120	300
10	LIDC-IDRI-0015	19	76	512 × 512	1.3	120	361
11	LIDC-IDRI-0016	26	104	512 × 512	2.5	120	265
12	LIDC-IDRI-0017	26	104	512 × 512	2.5	120	265

URL for download: https://cabig.nci.nih.gov/tools/NCIA.

**Table 2:** Performance comparison of the (MeQryEP) with other existing methods in terms of ARR on LIDC-IDRI-CT database.

	LBPu2	LBPriu2	LQP	DLTerQEP	LMeP	LMeTerP	LQEQryP	PM-MeQryEP
**ARR**	0.5717	0.6582	0.7654	0.803	0.8328	0.8572	0.8033	**0.9628**

Bold value is showing the best performance value by the proposed descriptor in the table. **Pm**: proposed method, i.e., MeQryEP.

**Table 3:** Data acquisition details of VIA/I-ELCAP-CT lung image database.

Data	No. of slices	Resolution	In-plane resolution	Slice thickness (mm)	Voltage (kv)
W1-10	100	512 × 512	0.76 × 0.76	1.25	120

URL for download: http://www.via.cornell.edu/-databases/lungdb.html.

**Table 4:** Group-wise performance of the proposed method and other existing methods in terms of recall values on VIA/I-ELCAP-CT database.

Method	LBPu2	LTP	LTCoP	LDP	LTrP	PVEP	LMeP	LMePu2	LQEP	LTrP	DLTerQEP	LQEQryP	PM-MeQryEP
Group													
1	32.44	36.05	38.4	37.73	33.03	36.03	37.43	37.18	38.23	33.03	42.39	42	42.42
2	40.5	34.87	36.03	37.14	36.85	39.85	35.45	34.7	34.78	36.85	36.02	39.75	40.88
3	38.67	39.11	38.99	45.59	43	40	28.9	30.5	38.76	43	41.72	41.58	43.9
4	66.95	59.94	70.01	61.49	62.4	63.4	72.97	73.07	65.79	62.4	70.12	72.2	73.9
5	36.17	32.11	39.67	32.64	41	40	37.93	36.55	40.29	41	41.6	44.42	45.07
6	54.24	48.09	53.22	46.61	51.7	59.7	52.9	50.63	54.15	51.7	54.72	63.94	64.22
7	48.49	36.54	49.45	38.4	51.4	52.4	53.27	48.57	52.08	51.4	52.66	58.89	58.97
8	81.18	78.24	84.23	77.11	89.5	91.5	95.56	85.57	88.79	89.5	88.14	94.17	95.08
9	47.84	43.11	46.09	44.24	41.9	48.9	42.96	42.04	43.11	41.9	44.65	47.59	48.9
10	72.67	67.19	68.57	68.55	69.55	78.55	69.58	72.03	68.08	69.55	68.63	69.93	72.74
Total	51.915	47.53	52.47	48.95	52.03	55.03	52.7	51.08	52.41	52.03	54.07	57.45	**58.61**

^*∗∗*^Bold value is showing the best performance value by the proposed descriptor in the table.

**Table 5:** MRI data acquisition details (adopted from [58]).

Sequence	MP-RAGE
TR (msec)	9.7
TE (msec)	4.0
Flip angle (o)	10
TI (msec)	20
TD (msec)	200
Orientation	Sagittal
Thickness, gap (mm)	1.25, 0
Resolution (pixels)	176 × 208

URL for download: http://www.ncbi.nlm.nih.gov/pubmed/17714011.

**Table 6:** Comparison of various techniques showing group-wise performance in terms of precision on the OASIS-MRI database.

Method	Precision (%) (*n* = 10)				
	Group 1	Group 2	Group 3	Group 4	Total
**LBPu2_8_1**	51.77	32.54	33.82	49.06	41.8
**CS_LBP**	44.7	40.1	31.17	48.27	41.06
**BLK_LBP**	48.13	41.22	35.16	50.01	43.63
**LTP**	56.53	36.27	34.97	50	44.44
**LDP**	46.29	36.37	36.82	45.56	41.26
**GLBPu2_8_1**	54.43	37.94	26.51	46.03	41.23
**LTrP**	49.55	36.99	35.45	47.01	42.25
**PVEP**	53.89	42.07	36.57	50.31	45.71
**LMePu2_8_1**	52.82	36.56	36.08	51.5	44.24
**LMEBP**	46.17	40.17	36.83	49.17	43.09
**LQEP**	50.97	36.37	39.1	35.57	40.5
**DLTerQEP**	54.27	42.65	37.08	46.42	45.11
**LMeTerP**	54.92	38.14	35.17	54.25	45.62
**LQEQryP**	54.11	43.04	36.74	51.04	46.23
**PM-MeQryEP**	54.84	43.02	36.13	53.12	46.78

Bold value is showing the best performance value by the proposed descriptor in the table.

**Table 7:** Feature vector length of query image using various methods.

Method	Feature vector length
LBP	256
LTP	2 × 256
LTCoP	2 × 256
LDP	4 × 256
LMeP	3 × 256
DLEP	4 × 512
LTrP	13 × 256
PVEP	4 × 256
LQEP	1 × 4096
LMeTerP	3 × 2 × 256
DLTerQEP	2 × 4096
LQEQryP	4 × 4096
PM-MeQryEP	3 × 4 × 256

## Data Availability

The data that support the findings of this study are available on reasonable request from the first author.

## References

[1] Schmidhuber J. (2015). Deep learning in neural networks: An overview. *Neural Networks*.

[2] Nanni L., Ghidoni S. (2017). How could a subcellular image, or a painting by Van Gogh, be similar to a great white shark or to a pizza?. *Pattern Recognition Letters*.

[3] Antani S., Long L. R., Thoma G. R. (2004). Content-based image retrieval for large biomedical image archives. *Proceeding of the 11th World Cong Medical Informatics*.

[4] Sihyoung L., Wesley D. N., Yong M. R. (2010). Tag refinement in an image folksonomy using visual similarity and tag co-occurrence statistics. *Signal Processing: Image Communication*.

[5] Yue G., Qionghai D., Meng W., Naiyao Z. (2011). 3D model retrieval using weighted bipartite graph matching. *Signal Processing: Image Communication*.

[6] Haralick R. M. (1979). Statistical and structural approaches to texture. *Proceedings of the IEEE*.

[7] Haralick R. M., Shanmugam K., Dinstein I. H. (1973). Textural features for image classification. *IEEE Transactions on Systems, Man, and Cybernetics*.

[8] Tamura H., Mori S., Yamawaki T. (1978). Textural features Corresponding to visual Perception. *IEEE Transactions on Systems, Man, and Cybernetics*.

[9] Roberti de Siqueira F., Robson Schwartz W., Pedrini H. (2013). Multi-scale gray level co-occurrence matrices for texture description. *Neurocomputing*.

[10] Verma M., Raman B., Murala S. (2015). Local extrema co-occurrence pattern for color and texture image retrieval. *Neurocomputing*.

[11] Do M. N., Vetterli M. (2002). Wavelet-based texture retrieval using generalized Gaussian density and Kullback-leibler distance. *IEEE Transactions on Image Processing*.

[12] Felipe J. C., Traina A. J. M., Traina C. J. Retrieval by content of medical images using texture for tissue identification.

[13] Jhanwar N., Chaudhuri S., Seetharaman G., Zavidovique B. (2004). Content based image retrieval using motif cooccurrence matrix. *Image and Vision Computing*.

[14] Liu W., Zhang H., Tong Q. (2008). Medical image retrieval based on nonlinear texture features. *Biomedical Engineering and Instrument Science*.

[15] Kassner A., Thornhill R. E. (2010). Texture analysis: a review of neurologic MR imaging applications. *American Journal of Neuroradiology*.

[16] Nanni L., Brahnam S., Ghidoni S., Menegatti E., Barrier T. (2013). Different Approaches for extracting information from the Co-occurrence matrix. *PLoS ONE*.

[17] Yadav K., Srivastava A., Mittal A., Ansari M. A. (2014). Texture-based medical image retrieval in compressed domain using compressive sensing. *International Journal of Bioinformatics Research and Applications*.

[18] Vaidehi K., Subashini T. S. (2015). An intelligent content based image retrieval system formammogram image analysis. *Journal of Engineering Science & Technology*.

[19] Ojala T., Pietikäinen M., Harwood D. (1996). A comparative study of texture measures with classification based on featured distributions. *Pattern Recognition*.

[20] Ojala T., Pietikainen M., Maenpaa T. (2002). Multiresolution gray-scale and rotation invariant texture classification with local binary patterns. *IEEE Transactions on Pattern Analysis and Machine Intelligence*.

[21] Takala V., Ahonen T., Pietikäinen M. (2005). Block-based methods for image retrieval using local binary patterns. *Image Analysis LNCS*.

[22] Heikkilä M., Pietikäinen M., Schmid C. (2009). Description of interest regions with local binary patterns. *Pattern Recognition*.

[23] Deep G., Kaur L., Gupta S. (2018a). Biomedical image retrieval using microscopicconfiguration with local structural information. *Sadhana*.

[24] Vipparthi S. K., Nagar S. K. (2014a). Expert image retrieval system using directional local motif XoR patterns. *Expert Systems with Applications*.

[25] Vipparthi S. K., Murala S., Nagar S. K., Gonde A. B. (2015b). Local Gabor maximum edge position octal patterns for image retrieval. *Neurocomputing*.

[26] Bala A., Kaur T. (2016). Local texton XOR patterns: A new feature descriptor for content-based image retrieval. *Engineering Science and Technology, an International Journal*.

[27] Nanni L., Lumini A. (2008a). Local binary patterns for a hybrid fingerprint matcher. *Pattern Recognition*.

[28] Zenghai C., Hui Z., Zheru C., Hong F. (2014). Hierarchical local binary pattern for branchretinal vein occlusion recognition. *ACCV Workshops, LNCS 9008*.

[29] Tan X., Triggs B. (2010). Enhanced local texture feature sets for face recognition under difficult lighting conditions. *IEEE Transactions on Image Processing*.

[30] Martolia M., Dhanore N., Singh A., Shahare V., Arora N. (2020). A modified local binary pattern (LBP) for content-based image retrieval. *International Journal of Advanced Science and Technology*.

[31] Murala S., Jonathan Wu Q. M. (2013a). Local ternary co-occurrence patterns: a new feature descriptor for MRI and CT image retrieval. *Neurocomputing*.

[32] Murala S., Jonathan W. Q. Peak valley edge patterns: a new descriptor for biomedical image indexing and retrieval.

[33] Murala S., Wu Q. M. J. (2014). Local mesh patterns versus local binary patterns: biomedical image indexing and retrieval. *IEEE Journal of Biomedical and Health Informatics*.

[34] Murala S., Maheshwari R. P., Balasubramanian R. (2012a). Directional binary wavelet patterns for biomedical image indexing and retrieval. *Journal of Medical Systems*.

[35] Murala S., Maheshwari R. P., Balasubramanian R. (2012b). Directional local extrema patterns: a new descriptor for content based image retrieval. *International Journal of Multimedia Information Retrieval*.

[36] Murala S., Maheshwari R. P., Balasubramanian R. (2012c). Local maximum edge binary patterns: a new descriptor for image retrieval and object tracking. *Signal Processing*.

[37] Murala S., Maheshwari R. P., Balasubramanian R. (2012d). Local Tetra patterns: A new feature descriptor for content-based image retrieval. *IEEE Transactions on Image Processing*.

[38] Koteswara Rao L., Venkata Rao D. (2015). Local quantized extrema patterns for content-based natural and texture image retrieval. *Human-centric Computing and Information Sciences*.

[39] Dubey S. R., Singh S. K., Singh R. K. (2015b). Local diagonal extrema pattern: a new and efficient feature descriptor for CT image retrieval. *IEEE Signal Processing Letters*.

[40] Vipparthi S. K., Murala S., Gonde A. B., Jonathan Wu Q. M. (2016). Local directional mask maximum edge patterns for image retrieval and face recognition. *IET Computer Vision*.

[41] Deep G., Kaur L., Gupta S. (2016a). Directional local ternary quantized extrema pattern: A new descriptor for biomedical image indexing and retrieval. *Engineering Science and Technology, an International Journal*.

[42] Deep G., Kaur L., Gupta S. (2016b). Local mesh ternary patterns: a new descriptor for MRI and CT biomedical image indexing and retrieval. *Computer Methods in Biomechanics and Biomedical Engineering: Imaging & Visualization*.

[43] Baochang Zhang B., Yongsheng Gao Y., Sanqiang Zhao S., Jianzhuang Liu J. (2010). Local derivative pattern versus local binary pattern: face recognition with high-order local pattern descriptor. *IEEE Transactions on Image Processing*.

[44] Nanni L., Lumini A., Brahnam S. (2010). Local binary patterns variants as texture descriptors for medical image analysis. *Artificial Intelligence in Medicine*.

[45] Paci M., Nanni L., Lahti A., Aalto-Setala K., Hyttinen J., Severi S. (2013). Non-binary coding for texture descriptors in Sub-Cellular and Stem Cell image classification. *Current Bioinformatics*.

[46] Vipparthi S. K., Nagar S. K. (2014). Color directional local quinary patterns for content based indexing and retrieval. *Human-Centric Computing and Information Sciences*.

[47] Nanni L., Paci M., Brahnam S., Ghidoni S. (2017). An ensemble of visual features for Gaussians of local descriptors and non-binary coding for texture descriptors. *Expert Systems with Applications*.

[48] Rampun A., Scotney B., Morrow P., Wang H., Winder J. (2018). Breast density classification using local quinary patterns with various Neighbourhood topologies. *Journal of Imaging*.

[49] Armi L., Fekri-Ershad S. (2019). Texture image Classification based on improved local Quinary patterns. *Multimedia Tools and Applications*.

[50] Rachdi E., Merabet Y. E., Akhtar Z., Messoussi R. (2020). Directional neighborhood topologies based multi-scale quinary pattern for texture classification. *IEEE Access*.

[51] Ahmad W., Shah S. M., Irtaza A. (2020). Plants disease phenotyping using quinary patterns as texture descriptor. *KSII Transactions on Internet and Information Systems*.

[52] Rubavathi C. Y., Ravi R. (2015). Local mesh co-occurrence pattern for content based image retrieval,” World Academy of Science. *Engineering and Technology (IJCEACIE)*.

[53] Zhu L., Zhang Y., Sun C., Yang andW. Face recognition with multiscale block local ternary patterns.

[54] Kascic E. (2011). *NBIA - National Cancer Imaging Archive NCIA (Version 4.0): The NCI’s Repository for DICOM-Based Images*.

[55] Nema-Ct (2012). NEMA-CT image database. http://ftp://medical.nema.org/medical/Dicom/Multiframe/.

[56] Lampert T., Stumpf A., Gancarski P. (2013). *An Empirical Study of Expert Agreement and Ground Truth Estimation*.

[57] Via/I-Elcap Ct (2003). VIA/I-ELCAP CT Lung Image Dataset. http://www.via.cornell.edu/-databases/lungdb.html.

[58] Marcus D. S., Wang T. H., Parker J., Csernansky J. G., Morris J. C., Buckner R. L. (2007). Open Access series of imaging studies (OASIS): cross-sectional MRI data in Young, Middle Aged, Nondemented, and Demented Older Adults. *Journal of Cognitive Neuroscience*.

